# A robust technique based on VLM and Frangi filter for retinal vessel extraction and denoising

**DOI:** 10.1371/journal.pone.0192203

**Published:** 2018-02-12

**Authors:** Khan Bahadar Khan, Amir. A. Khaliq, Abdul Jalil, Muhammad Shahid

**Affiliations:** 1 Department of Telecommunication Engineering, The Islamia University Bahawalpur, Pakistan; 2 Department of Electronic Engineering, International Islamic University, Islamabad, Pakistan; 3 Al-Khawarizmi Institute of Computer Science, UET Lahore, Pakistan; University of California Santa Barbara, UNITED STATES

## Abstract

The exploration of retinal vessel structure is colossally important on account of numerous diseases including stroke, Diabetic Retinopathy (DR) and coronary heart diseases, which can damage the retinal vessel structure. The retinal vascular network is very hard to be extracted due to its spreading and diminishing geometry and contrast variation in an image. The proposed technique consists of unique parallel processes for denoising and extraction of blood vessels in retinal images. In the preprocessing section, an adaptive histogram equalization enhances dissimilarity between the vessels and the background and morphological top-hat filters are employed to eliminate macula and optic disc, etc. To remove local noise, the difference of images is computed from the top-hat filtered image and the high-boost filtered image. Frangi filter is applied at multi scale for the enhancement of vessels possessing diverse widths. Segmentation is performed by using improved Otsu thresholding on the high-boost filtered image and Frangi’s enhanced image, separately. In the postprocessing steps, a Vessel Location Map (VLM) is extracted by using raster to vector transformation. Postprocessing steps are employed in a novel way to reject misclassified vessel pixels. The final segmented image is obtained by using pixel-by-pixel AND operation between VLM and Frangi output image. The method has been rigorously analyzed on the STARE, DRIVE and HRF datasets.

## Introduction

The fundamental target of retinal vessel segmentation is to investigate the existence of DR conditions, being a noteworthy reason for visual deficiency in working age people in the United States [1]. The major observed signs of DR comprise hemorrhages, dilated retinal veins, cotton wool spots and hard exudates [2]. Disparities in retinal vascular features are signs of severe ailments, such as diabetes, stroke and cardiovascular diseases [3]. Retinal vascular changes are irretrievable, even restoration technique would not help the patient to have the same vision capability as was before the disease. Therefore, the timely detection of DR from a fundus camera image will protect the enduring person from having an irreversible visual deficiency.

Segmentation is an essentially basic step of the retinal disorders identification in the medical imaging domain. The premature stages of hypertension, cardiovascular ailment, diabetes, arteriosclerosis and stroke can be traced by a comprehensive investigation of the retinal vessel network [4]. It gives an opportunity to the patient to take an action against the infection before it reaches to its climax. Moreover, it has been used to distinguish miscellaneous things in the retina image. The segmentation of an object or substance is based on discrimination with respect to edges, shape and correlation with the background in an image. Currently, the deep or the hierarchical features are utilized for segmentation of the image. These features are too numerous and computationally expensive to use them for critical time applications. These deep features, however, produce good results. Segmentation strategies attempt to locate boundaries and interrelated segments in the photographs and add shape’s information to detain the succeeding state segmentation [5].

Ophthalmologist use fundus camera and Optical Coherence Tomography (OCT) images to scrutinize the retina and its inside sectors containing vessels’ network, fovea, optic disk and so on [6]. Retinal vasculature offers useful information to numerous disease monitoring applications, including recuperative analysis and categorization of ophthalmological disorders and cardiovascular diseases. The vessel tree can be used to expose the hypertensive retinopathy along with an approximation of vessels breadth, which is incorporated to investigate hypertension [7]. The DR can be perceived by variations in the vasculature spreading [6]. Moreover, vessels segmentation is used to help laser surgical procedures [8] and as a revolutionary technique for image registration [9]. The vessel tree delineation in retina image is an essential preprocessing step for all above mentioned operations.

The retinal vessel identification is a difficult task on account of poor contrast and correlated geometrical abnormalities in the background of an image. A strong image processing, computer vision and machine learning tools are required to perform this task. There are numerous issues with the current retinal vessel segmentation methods: some of them are manual, semi-automated and others are automated, some methods have time complexity and some suffer from degradation in accuracy with the change of the dataset. The purpose of blood vessel segmentation is to extract complete vessel structure while eliminating all other geometric objects like macula, optic disc and other retinal abnormalities.

The fundamental target of the current research is to propose an automatic retinal blood vessels segmentation technique employing computationally less hungry tools of image processing and computer vision. There are various image processing procedures which can produce good results but are computationally expensive. In this study, a robust and time efficient method has been suggested. In the proposed method, a combination of different preprocessing, enhancement, segmentation and postprocessing techniques have been employed. The pursuance of segmentation method has been rigorously studied by performance metrics like accuracy (Acc), Sensitivity (Sn), Specificity (Sp) and ROC curve on the typical datasets like DRIVE, STARE and HRF.

This article is structured into five sections: Introduction (Sect. 1), Related Literature (Sect. 2), Proposed Model (Sect. 3), Experimental analysis and Discussion (Sect. 4) and the conclusion (Sect. 5).

## Related literature

The automated delineation of retinal vasculature is a preliminary task in the field of computer-aided identification. Therefore, the worth of vessel segmentation technique is immensely influential in the development of retinal disease diagnosis. A technique that can be built up to help in deduction of DR or any other ocular disease have to differentiate all kinds of landscapes in the retinal image, for instance, optic disk, blood vessels, fovea and all other abnormalities due to diseases, including cotton wool spots, hemorrhages, microaneurysms and edema [10].

The retinal vessel map in fundus image can be delineated by numerous vessel extraction procedures that have already been published in the literature [10–11]. The vessel detection approaches can usually be sorted into two groups: supervised and unsupervised classification, based on machine learning procedures. Supervised classification method isolates the foreground and background pixels using neighboring pixel based feature vectors to train a classifier. Whereas, there is no need of training a classifier in unsupervised strategies [12]. Generally, the supervised methods are time consuming as compared to unsupervised methods. Therefore, a small number of research papers are presented in the literature using this strategy.

Supervised classification methods comprise training and testing phase. In training phase, it requires a ground truth image produced by an expert in that field to learn features. These learned features are used for classification purpose in testing phase. Niemeijer et al. [13] used green channel for feature array abstraction of every pixel and k-Nearest Neighbor (kNN) classifier has been utilized to isolate foreground and background retinal pixels. Staal et al. [14] suggested a technique based on the abstraction of image ridges to extract retinal vessel network, which correspond roughly with vessel midlines. The characteristic vectors are grouped making use of kNN and succeeding onward feature choice. Soares et al. [15] used pixel’s luminosity to take feature array and 2D Gabor transform has been applied to isolate True Positive (TP) and False Positive (FP) retinal pixels and lastly delineation by utilizing a Gaussian Mixture Model (GMM). Support Vector Machine (SVM) is utilized to acquire a feature vectors recommended by Ricci et al. [16]. The SVM is further utilized by Xu & Luo [17] to segregate vessel and background pixels, followed by tracking growth approach to extract the thin vessel pixels and to obtain final binary image. You et al. [18] introduced a radial projection based approach to detect midlines of the vessels, focusing on tiny and low resolution vessels coupling with semi-supervised self-training scheme for recognition of wide vessels. The combination of these techniques produced a resultant binary image. In [19], a number of concavity modeling practices has been utilized for blood vessel dissection. Bright lacerations are controlled by differentiable concavity extent; dark lesions are detached and eliminated by using line-shape concavity; and random noise is accomplished by local normalized concavity measure. These concavity extent quantities are fused together based on their statistical scatterings to discriminate foreground and background pixels. Joshi et al. [20] used a graph search process for exposure and isolation of retinal vessel tree using a supervised automated technique. A novel three steps approach for detection of retinal binary vessels map is presented by Roychowdhury et al. [21]. In the preliminary step, a major vessel network is obtained by coupling the two binary images from high pass filtering and from morphological reconstruction, respectively. In the 2^nd^ step, the residual pixels are categorized by GMM. In the final step, the major segments of vessels are coupled with the categorized vessel pixels. Liskowski & Krawiec [22], proposed a deep neural network approach for delineation of retinal vascular network. Recently, a discriminatively trained fully-connected Conditional Random Field (CRF) approach is proposed for segmentation of retinal vasculature [23].

In contrast to a supervised method, the unsupervised techniques achieve the delineation of vessels in retina image without incorporating trained material or any grouping methods. Most of the segmentation techniques in literature belong to this class as it is computationally less expensive. Chaudhuri et al. [24] designed a 2D matched filter with the help of a Gaussian shaped curvature to extract retinal vascular tree. Hoover et al. [25] utilized local and global vessel features equally by putting on a Matched Filter Response (MFR) and thresholding to fragment the vessel tree. Zana and Klein [26] used the cross-curvature assessment and morphological operations collectively for vessel segmentation but their suggested framework was not capable to delineate the thinner vessels properly. Mendonca and Campilho [27] employed the responses of differential filters along with morphological filter for the recognition of centerline of vessel, vessel features and morphological features for filling the vascular. Matinez-Perez et al. [28] has incorporated 1^st^ and 2^nd^ order spatial derivatives of the pixel intensity that provide specific vessel structure to control the intrinsic problem of contrast deviations in fundus photographs. This procedure also allows the investigation of variation in vessels orientations, elongated structure and diameter. In [29], a vigorous contouring model is presented for vessels border detection and tolerate to vessel width uniformity. Palomera-Pérez et al. [30] proposed technique utilized multi-level feature creation and region growing technique for retinal vessel identification. Lupaşcu et al. [31] has incorporated Self Organizing Map (SOM) and K-means grouping procedure for training and discovering of vessel map. Hill ascending policy is utilized for further processing of binarized image. Centerline recognition procedures and morphological based bit plane model for vessel tree segregation have been used by Fraz et al. [32]. In [33], wavelets transformation and edge position based boosting method for vessel tree segmentation has been used. Zhao et al. [34] employed an efficient graph cut scheme with retinex and local phase based method and produced promising results. Dai et al. [35] introduced a gray-voting and GMM classifier based approach for detection of retinal vessel network. A new region-based active contour model is presented by introducing a novel multi-feature Gaussian distribution fitting energy model [36]. Oliveira et al. [37] used combined MF, Frangi’s filter and Gabor wavelet filter to improve the photographs contrast, followed by deformable models and the fuzzy C-means for retinal vessels extraction. Khan et al. [38] proposed a morphological Hessian based technique followed by Otsu thresholding for recognition of retinal vascular map. Lázár and Hajdu [39] suggested a region growing technique for segmentation of retinal vessels which coupled a hysteresis thresholding arrangement with the response vector resemblance of neighboring pixels. A multiscale graph-based retinal vessel extraction is performed by utilizing some of perceptual Gestalt principles [40]. Singh and Srivastava [41] introduced a combination of Gumbel PDF based MF, entropy based optimal thresholding, region based filtering and eradicating isolated objects by utilizing the perception of masking.

## Proposed model

This section demonstrates a proposed way to enhance and segment blood vessels in retina images. Two parallel processes for noise elimination and vasculature based enhancement have been employed. The main target of this work is to effectively eradicate noise and other diseases’ abnormalities which are often enhanced and appeared as vessel pixels in case of simple enhancement techniques. Such noise and disorders have been removed by extracting VLM separately, which is coupled by AND operation with the binary output of the Frangi filter applied for vascular enhancement, separately. The flowchart of the suggested segmentation procedure is portrayed in Fig 1 and its detailed steps are given below.

**Fig 1:** Step-wise illustration of the proposed system.

- Green band is extracted from the RGB input retinal photograph due to its prominent vascular contrast.
- Mask creation from red channel to extract a Region Of Interest (ROI).
- Image contrast enhancement performed by Contrast Limited Adaptive Histogram Equalization (CLAHE) and morphological filters have been utilized to eradicate low frequency noise/entities like optic disc, macula, etc.
- High boost filter has been applied to enhance the edges of thick vessels and to enhance thin vessels from the background. It is high pass filtering operation.
- Frangi filter has been employed for vascular based enhancement.
- Improved Otsu based thresholding has been used on the high boost filtered image and Frangi filter enhanced image to find optimal threshold value, followed by hysteresis thresholding for image binarization.
- Postprocessing steps have been used to compute area and eccentricity based threshold, which is further utilized to extract a final VLM.
- The pixel-by-pixel AND operation has been applied between already binarized images to acquire final image.

### Preprocessing steps

Vessel segmentation in retina image becomes a really complicated task especially in pathological cases due to colossal contrast variation, vessel like abnormal structures and vessel leakage due to diseases. Pixel intensity transformation has been applied for the purpose of vessel enhancement from the background. There are many Histogram Equalization (HE) methods for contrast enhancement like global HE and local HE. The HE [42], uses probability density based transformation function for adjustment of intensity values. In histogram equalization, each intensity value is mapped to a new value based on well-defined neighboring pixel values, e.g. in local contrast enhancement pixel values within defined window is used for transformation function. Adaptive Histogram Equalization (AHE) is a famous contrast enhancement approach for health and natural image modalities suggested by Pizer [43].

The CLAHE [44] is an innovative version of AHE known as fairly fast with good confined contrast results. CLAHE was primarily aimed for enhancement of having a small gap between foreground and background medical images [45]. CLAHE is different as compared to usual AHE in limiting the contrast enhancement. CLAHE takes a user-given rate known as clip limit to bound enhancement by trimming the histogram [44]. The clipping limit identifies that the noise level should be flattened and gap between vessels and non-vessels to be increased.

Red channel is an excellent candidate for mask creation as it has a good contrast between the background and the foreground. A mask has been created to confine the computation within the ROI. Modified top-hat image is obtained using Open and Close morphological filters. Finally, the high boost filter has been employed to enhance the edges of wide vessels and enhance thin vessels from the background.

### Frangi filter based vascular enhancement

Frangi filter employs Hessian eigenvalues based approach on the high boost filtered image for the vessel contrast enhancement along with suppression of non-vascular structure of wide and thin vessels. The Hessian matrix is computed by manipulative the 2nd order derivative of an image in x-axis, y-axis and both left and right diagonals.

A vessel detection filter based on Hessian can be described as

$$F(x)={max}_{\sigma \;}f(x,\sigma )$$ (1)

where *x* is a location of pixel in an image; *f* is the filter utilized for vessel detection and *σ* is the standard deviation for computing Gaussian image derivative.

The vessel direction is aligned along the x-axis by rotating the coordinates to reduce the noise sensitivity of the Hessian eigenvalues based approach. Suppose the directional image *I*_*i*_ (*i* = 1, …, *n*) corresponds to the orientations ranging from *θ*_*i*_,_*min*_ to *θ*_*i*,*max*_ (counterclockwise angle). Its associated coordinates *C*xy will be rotated to *C x*′*y*′ by an amount as large as the mean value *θ*_*i*_

$$\theta_{i}=\frac{\theta_{i,min}+\theta_{i,max}}{2}$$ (2)

Hessian matrix of the directional image *I*_*i*_ in the new coordinates *C x*′*y*′ is computed as [46]

$$H^{\prime }=\left[\begin{array}{cc} h_{11} & h_{12}\\ h_{21} & h_{22} \end{array}\right]=\left[\begin{array}{cc} \frac{\partial^{2}I_{i}}{\partial {x^{\prime }}^{2}} & \frac{\partial^{2}I_{i}}{\partial x^{\prime }\partial y^{\prime }}\\ \frac{\partial^{2}I_{i}}{\partial y^{\prime }\partial x^{\prime }} & \frac{\partial^{2}I_{i}}{\partial {y^{\prime }}^{2}} \end{array}\right]$$ (3)

where

$$\frac{\partial^{2}I_{i}}{\partial {x'}^{2}}=\frac{\partial^{2}I_{i}}{\partial x^{2}}{cos}^{2}\theta_{i}+\frac{\partial^{2}I_{i}}{\partial x\partial y}\text{sin}(2\theta_{i})+\frac{\partial^{2}I_{i}}{\partial y^{2}}{sin}^{2}\theta_{i}$$ (4)

$$\frac{\partial^{2}I_{i}}{\partial {y'}^{2}}=\frac{\partial^{2}I_{i}}{\partial x^{2}}{sin}^{2}\theta_{i}-\frac{\partial^{2}I_{i}}{\partial x\partial y}\text{sin}(2\theta_{i})+\frac{\partial^{2}I_{i}}{\partial y^{2}}{cos}^{2}\theta_{i}$$ (5)

$$\frac{\partial^{2}I_{i}}{\partial {x'}^{}\partial {y'}^{}}=\frac{\partial^{2}I_{i}}{\partial {y'}^{}\partial {x'}^{}}=-\frac{1}{2}\frac{\partial^{2}I_{i}}{\partial x^{2}}\text{sin}(2\theta_{i})+\frac{\partial^{2}I_{i}}{\partial x\partial y}\text{cos}(2\theta_{i})+\frac{1}{2}\frac{\partial^{2}I_{i}}{\partial y^{2}}\text{sin}(2\theta_{i})$$ (6)

where *h*_11_, *h*_12_, *h*_21_, and *h*_22_ are the directional 2^nd^ order partial derivatives of the image. The eigenvalues transformation has been applied on Hessian matrix to acquire eigenvalues *λ*_1_ and *λ*_2_ to decide the likelihood of *x* belonging to a vessel, while *σ* is utilized to describe the scale of vessel enhancement. The filter response will be ideal, if the scale *σ* matches the size of the vessel. The exploration is based on the below assumption:

$$\left|\lambda_{1}|\leq |\lambda_{2}\right|$$

f(x,σ)=0,

where *λ*_2_ > 0

$${{h'}^{}}_{11}=\sigma^{2}*h_{11}$$ (7)

$${{h'}^{}}_{12}={{h'}^{}}_{21}=\sigma^{2}*h_{12}$$ (8)

$${{h'}^{}}_{22}=\sigma^{2}*h_{22}$$ (9)

$$R_{B}=\lambda_{1}/\lambda_{2}$$ (10)

$$S=\surd ({\lambda_{1}}^{2}+{\lambda_{2}}^{2})$$ (11)

$$\begin{array}{cc} I_{E}= & \{\begin{array}{ll} 0, & if\;\lambda_{2}>0,\\ exp\left(-R_{B}^{2}/2\beta^{2}\right) & \left(1-exp\left(\frac{-S^{2}}{2c^{2}}\right)\right) \end{array} \end{array}$$ (12)

where *c* and β are constants which control the sensitivity of filter. *S* can be computed from Eq 11. where *R*_*B*_ is used with β to discriminate plain line like structures from blob like structures and *S* is used with *c* for eliminating background noise. *c* and β are the are the parameters controlling *R*_*B*_ and *S*. The complete shape judgment and noise eradication is reliant on the values of *c* and β. Enhanced Image *I*_*E*_ is obtained at different scales using values 1.5 and 4.5 for *σ* in Eqs 7–9. Histogram based visual representation of the applied preprocessing contrast enhancement schemes is shown in Fig 2. The pictorial analysis of thin and wide vessels enhancement using Frangi filtering method on the DRIVE and STARE datasets are shown in Figs 3 and 4, respectively.

**Fig 2:** Histogram based visual representation of the applied preprocessing contrast enhancement schemes. (a) Green channel image (b) CLAHE (c) TopHat image (d) Frangi enhanced image.

**Fig 3:** Analysis of Frangi filtering enhancement using DRIVE dataset. (a) Thin vessel enhanced image (b) Thin binary image (c) Thick vessel enhanced image (d) Thick binary image.

**Fig 4:** Analysis of Frangi filtering enhancement using STARE dataset. **A** (a) Thin vessel enhanced image (b) Thin binary image (c) Thick vessel enhanced image (d) Thick binary image.

### Improved Otsu thresholding

A 2D gray level intensity function *f*(*x*, *y*) is used to symbolize an input picture with dimension *M* x *N*, where 0 ≤ *f*(*x*, *y*) ≤ *L* − 1 and L represents the number of distinct gray levels. The gray level of a pixel and its local average both are utilized in a 2D thresholding technique [47]. The function of the local average *g*(*x*, *y*) is used to symbolize the local average gray level which is also distributed into the similar L values and is given by

$$g\left(x,y\right)=\frac{1}{n^{2}}\sum_{m=-l/2}^{i=l/2}\sum_{n=-l/2}^{j=l/2}f\left(x+m,y+n\right)$$ (13)

where *l* ≤ min{*M*, *N*}. The variable M and N represent an input picture with dimension M x N.

Let *t*_*mn*_ be the over-all numeral of incidence of the couple (*m*, *n*), which symbolizes pixel (*x*, *y*) with *f*(*x*, *y*) = *m* and *g*(*x*, *y*) = *n*, 0 ≤ *t*_*mn*_ ≤ *M* x *N*, then the joint probability mass function *p*_*mn*_ is known by

$$p_{mn}=\frac{t_{mn}}{M\;\text{x}\;N}$$ (14)

where $m,n=0,\ldots \;\ldots ,L-1,\sum_{m=0}^{L-1}\sum_{n=0}^{L-1}p_{mn}=1.$

The 2D histogram of the picture is {*p*_*mn*_}. Fig 5 displays the top view of 2D histogram. It represents a square area with dimension *L* x *L*. The 2D histogram is partitioned into four quadrants at an array (*S*, *T*), where 0 ≤ *S*, *T* ≤ *L* − 1. The dotted track in the center is the diagonal of 2D histogram. The pixels interior to the objects or the background should contribute mostly to the near-diagonal components due to similarity. Because, the gray level of a pixel and its local average are similar for the pixels inside to the objects and background, where it is dissimilar for the pixels in the neighborhood of an edge between the objects and the background. Consequently, quadrants A and C consist the spreading of object and background clusters, whereas the off-diagonal quadrants B and D consist the distributions of pixels adjacent boundaries and noises.

**Fig 5:** 2D histogram top view.

Now assume that the pixels are segregated into two clusters *C*_0_ and *C*_1_ (background and objects) by a threshold pair (*s*, *t*), then the occurrences of two clusters are assumed by [47]

$$P_{0}\left(s,t\right)=\sum_{m=0}^{s}\sum_{n=0}^{t}p_{mn}$$ (15)

$$P_{1}\left(s,t\right)=\sum_{m=s+1}^{L-1}\sum_{n=t+1}^{L-1}p_{mn}$$ (16)

The mean of two clusters are given by

$$\mu_{0}={\left(\mu_{00},\mu_{01}\right)}^{T}={\left(\sum_{m=0}^{s}\sum_{n=0}^{t}m.p_{mn}/P_{0},\sum_{m=0}^{s}\sum_{n=0}^{t}n.p_{mn}/P_{0}\right)}^{T}$$ (17)

$$\mu_{1}={\left(\mu_{10},\mu_{11}\right)}^{T}={\left(\sum_{m=s+1}^{L-1}\sum_{n=t+1}^{L-1}m.p_{mn}/P_{1},\sum_{m=s+1}^{L-1}\sum_{n=t+1}^{L-1}n.p_{mn}/P_{1}\right)}^{T}$$ (18)

The total mean vector is

$$\mu_{T}={\left(\mu_{T0},\mu_{T1}\right)}^{T}={\left(\sum_{m=0}^{L-1}\sum_{n=0}^{L-1}m.p_{mn},\sum_{m=0}^{L-1}\sum_{n=0}^{L-1}n.p_{mn}\right)}^{T}$$ (19)

Generally, the probability of the off-diagonal image data can be negligible. So, it is easy to be confirmed that

$$P_{0}+P_{1}=1,\mu_{T}\approx P_{0}\mu_{0}+{P_{1}\mu }_{1}$$ (20)

The between-class variance matrix is given as

$$S_{B}=\sum_{k=0}^{1}P_{k}[(\mu_{k}-\mu_{T}){\left(\mu_{k}-\mu_{T}\right)}^{T}]$$ (21)

By utilizing the trace of *S*_*B*_ as the between class variance can be computed as

$$t_{r}S_{B}=P_{0}[{\left(\mu_{00}-\mu_{T0}\right)}^{2}+{\left(\mu_{01}-\mu_{T1}\right)}^{2}]+P_{1}[{\left(\mu_{10}-\mu_{T0}\right)}^{2}+{\left(\mu_{11}-\mu_{T1}\right)}^{2}]=\frac{{\left(\mu_{m}\left(s,t\right)-P_{0}\mu_{T0}\right)}^{2}+{\left(\mu_{n}\left(s,t\right)-P_{0}\mu_{T1}\right)}^{2}}{P_{0}\left(1-P_{0}\right)}$$ (22)

where

$$\mu_{m}\left(s,t\right)=\sum_{m=0}^{s}\sum_{n=0}^{t}m.p_{mn}$$

$$\mu_{n}\left(s,t\right)=\sum_{m=0}^{s}\sum_{n=0}^{t}n.p_{mn}$$

The optimal threshold is the threshold that maximize *t*_*r*_*S*_*B*_.

### Postprocessing steps

The discrete steps in postprocessing are shown in Fig 6. Before applying these postprocessing steps, a few unconnected pixel’s patch and salt noise has been removed to save time and computational cost. In the preliminary step, a raster to vector transformation has been applied for individual unconnected patch labeling. The physical properties i.e. eccentricity and area of each labeled patch or vector has been computed. As the vessels are connected and elongated patches, therefore, they have the higher area and eccentricity (length, width ratio) almost equal to one. Area tells about the total number of connected pixels in a segment while eccentricity shows the ratio of length and width (elongation). The vessels are elongated and connected in nature and having large number of pixels. So, high value of area and eccentricity tells us about the presence of vessels. The segments which have less value of area (less than 250 pixels) and eccentricity (0.95) are clipped. A threshold limit has been selected based on these physical properties for noisy segments rejection. The pixel-by-pixel AND operation has been applied between already binarized images to acquire final image. Fig 7 validates that if we used another operator like OR operator it will again add noise which is trimmed in noise elimination stage.

**Fig 6:** Steps for extraction of VLM.

**Fig 7:** Analysis of using OR operator. (a) RGB input image (b) VLM (c) Frangi enhanced, thresholded image (d) OR Operator result.

Pictorial effects of principal processing stages of the planned procedure for vessel segmentation using the STARE [25] [S1 File], DRIVE [14] [S2 File] and HRF [48][S3 File] datasets are revealed in Figs 8, 9 and 10, correspondingly. The VLM is an innovative approach to produce good visual and quantitative results. In this approach, the background noise removal and vessel enhancement have been performed separately.

**Fig 8:** Visual presentation of the proposed system major processing stages. (a) Input RGB photograph from **STARE** database (b) Green channel (c) CLAHE applied result (d) Difference image (e) Otsu threshold resultant image (f) Postprocessed dilated image (g) Frangi filter enhanced image (h) Final image using AND Operation.

**Fig 9:** Visual presentation of the proposed system major processing stages. (a) Input RGB photograph from **DRIVE** database (b) Green channel (c) CLAHE applied result (d) Difference image (e) Otsu threshold resultant image (f) Postprocessed dilated image (g) Frangi filter enhanced image (h) Final image using AND Operation.

**Fig 10:** Visual presentation of the Proposed system major processing stages. (a) Input RGB photograph from **HRF** database (b) Green channel (c) CLAHE applied result (d) Difference image (e) Otsu threshold resultant image (f) Postprocessed dilated image (g) Frangi filter enhanced image (h) Final image using AND Operation.

## Experimental analysis and discussion

In this section, the details about datasets, performance validation criteria, experimental results and discussion, VLM analysis and time computation analysis are discussed.

### Datasets

The success of the proposed methodology has been measured and compared with recent frameworks on the three freely accessible datasets: STARE [25], DRIVE [14] and HRF [48]. The DRIVE and STARE databases comprise of 20 and 40 fundus photographs, correspondingly divided into two groups: training part and test part. In both datasets, the segmentation produced by first grader has been engaged as a gold standard for assessment, whereas the segmentation of second grader has been used for performance analysis. The HRF datasets consist of 45 images divided into three different groups: 15 normal retina images, 15 images of patients with DR and 15 images of glaucomatous patients. Binary ground truth data for each image is provided in the dataset. The accuracy, specificity and sensitivity parameters are used for performance evaluation criteria of the proposed system with other existing frameworks.

### Performance assessment measures

The performance measures for detection of retinal vessel network are exposed in Table 1.

**Table 1:** Performance metrics for evaluation of the proposed method.

Metrics	Explanation
True Positive Rate (TPR)	TP/vessel pixel count
False Positive Rate (FPR)	FP/non-vessel pixel count
Sensitivity(Sn)	TPR or TP/(TP+FN)
Specificity(Sp)	1-FPR or TN/(TN+FP)
Accuracy(Acc)	(TP+TN)/(TP+FP+TN+FN)
Area under the ROC curve (AUC)	Sn+Sp/2

Where TP, TN, FP and FN represent the True Positive (precisely spotted vessel pixels), True Negative (correctly perceived non-vessel pixels), False Positive (erroneously recognized vessel pixels) and False Negative (imperfectly detected non-vessel pixels), correspondingly. Sensitivity shows the ability of the algorithm to accurately identify blood vessels, while specificity demonstrates the competence of discovering all other non-vessel segments. Accuracy exhibits overall system performance, while AUC reflect the trade-offs between the sensitivity and specificity.

### Results and analysis

Table 2 shows that the effectiveness of the proposed system has been confirmed on three openly accessible datasets: DRIVE, STARE and HRF. The average accuracy for the STARE database is 0.951, for the DRIVE database is 0.958 and 0.952 for HRF dataset. The proposed technique has produced maximum possible accuracy with average sensitivity on both datasets. Manual segmentation done by a human grader is also incorporated into the assessment. Table 3 shows that the proposed method has acquired a good accuracy as contested to many other approaches in the literature.

**Table 2:** Accuracy (Acc), Sensitivity (Sn) and Specificity (Sp) statistics of the proposed system on the DRIVE, STARE and HRF databases.

Images	DRIVE			STARE			HRF		
	Acc	Sn	Sp	Acc	Sn	Sp	Acc	Sn	Sp
1	0.956	0.798	0.971	0.940	0.716	0.960	0.950	0.702	0.976
2	0.961	0.808	0.978	0.951	0.625	0.974	0.943	0.801	0.950
3	0.958	0.625	0.991	0.930	0.793	0.939	0.965	0.741	0.978
4	0.962	0.670	0.989	0.956	0.757	0.972	0.959	0.721	0.964
5	0.967	0.732	0.988	0.952	0.747	0.973	0.944	0.650	0.958
6	0.953	0.658	0.983	0.963	0.770	0.978	0.957	0.710	0.962
7	0.957	0.796	0.970	0.944	0.887	0.949	0.956	0.771	0.952
8	0.952	0.768	0.966	0.950	0.872	0.956	0.952	0.750	0.965
9	0.958	0.651	0.985	0.944	0.868	0.951	0.945	0.730	0.976
10	0.963	0.771	0.978	0.949	0.829	0.960	0.963	0.770	0.964
11	0.958	0.717	0.979	0.951	0.819	0.961	0.958	0.745	0.975
12	0.959	0.766	0.976	0.954	0.892	0.959	0.941	0.715	0.972
13	0.952	0.689	0.982	0.950	0.820	0.963	0.951	0.734	0.958
14	0.960	0.795	0.973	0.950	0.826	0.963	0.959	0.751	0.948
15	0.946	0.772	0.960	0.947	0.829	0.958	0.949	0.809	0.947
16	0.961	0.755	0.980	0.946	0.718	0.972	0.948	0.726	0.957
17	0.961	0.771	0.976	0.953	0.816	0.966	0.945	0.732	0.935
18	0.962	0.715	0.987	0.976	0.704	0.991	0.953	0.805	0.924
19	0.958	0.682	0.989	0.963	0.832	0.969	0.956	0.760	0.947
20	0.954	0.663	0.984	0.956	0.684	0.975	0.952	0.781	0.959
**Average**	**0.958**	**0.730**	**0.9793**	**0.9513**	**0.7902**	**0.9645**	**0.9523**	**0.7452**	**0.9584**

**Table 3:** Performance evaluations of various retinal vascular extraction algorithms.

Technique	Year	DRIVE				STARE			
		Acc	Sn	Sp	AUC	Acc	Sn	Sp	AUC
Human observer		0.947	0.776	0.972	0.874	0.935	0.895	0.939	0.917
Unsupervised techniques									
Zana and Klein [26]	2001	0.938	0.697	—	—	—	—	—	—
Mendonça [27]	2006	0.945	0.734	0.976	0.855	0.944	0.699	0.973	0.836
Martinez-Perez [28]	2007	0.934	0.725	0.965	0.845	0.941	0.751	0.955	0.853
Al-Diri [29]	2009	—	0.728	0.955	0.842	—	0.752	0.968	0.860
Palomera-Perez [30]	2010	0.922	0.660	0.961	0.811	0.924	0.779	0.940	0.860
Lupaşcu [31]	2010	0.946	0.696	0.970	0.833	—	—	—	—
Fraz [32]	2012	0.943	0.715	0.976	0.845	0.944	0.731	0.968	0.850
Bankhead [33]	2012	0.937	0.703	0.971	0.837	0.932	0.758	0.950	0.854
Zhao [34]	2015	0.953	0.744	0.978	0.861	0.951	0.786	0.975	0.881
Dai [35]	2015	0.942	0.736	0.972	0.854	0.936	0.777	0.955	0.866
Wang [36]	2015	—	—	—	—	0.944	0.758	0.965	0.862
Lázár [39]	2015	0.946	0.765	0.972	0.869	0.949	0.725	0.975	0.850
Oliveira [37]	2016	0.946	0.864	0.956	0.910	0.953	0.825	0.965	0.895
Khan [38]	2016	0.961	0.746	0.980	0.863	0.946	0.758	0.963	0.861
Al Shehhi [40]	2016	0.934	0.850	0.944	0.897	0.924	0.633	0.950	0.792
Singh [41]	2016	0.952	0.759	0.971	0.865	0.927	0.794	0.938	0.866
**Proposed**	**2016**	**0.958**	**0.730**	**0.979**	0.855	**0.951**	**0.790**	**0.965**	**0.878**
Supervised techniques									
Niemeijer [13]	2004	0.942	0.690	0.970	0.830	—	—	—	—
Staal [14]	2004	0.944	0.719	0.977	0.848	0.952	0.697	0.981	0.839
Soares [15]	2006	0.946	0.724	0.976	0.850	0.948	0.710	0.974	0.842
Xu and Luo [17]	2010	0.933	0.776	—	—	—	—	—	—
Lam [19]	2010	0.947	—	—	—	0.957	—	—	—
You [18]	2011	0.943	0.741	0.975	0.858	0.950	0.726	0.976	0.851
Roychowdhury [21]	2015	0.952	0.725	0.983	0.854	0.951	0.772	0.973	0.873
Orlando [23]	2016	0.945	0.790	0.968	0.879	0.957	0.777	0.979	0.878

In Table 3, the Acc, Sn and Sp values of Xu and Luo [17], Lam [19], You [18], Roychowdhury [21], Orlando [23], Martinez-Perez [28], Al-Diri [29], Palomera-Perez [30], Lupaşcu and Tegolo [31], Fraz [32], Bankhead [33], Zhao [34], Dai [35], Wang [36], Lázár and Hajdu [39], Oliveira [37], Khan [38], Al Shehhi [40] and Singh and Srivastava [41] are achieved from their published papers, while Staal [14] and Soares [15] results are acquired from their websites. The results of Zana and Klein [26] method were performed by Niemeijer [13]. The AUC results of all methods in Table 3 are calculated using the formula mentioned in Table 1. The proposed model has achieved the highest accuracy on the DRIVE database among all other supervised and unspervised approaches except Khan [38] method which is 0.003 better comparatively. On the STARE database, accuracy of Oliveira [37], Staal [14], Lam [19] and Orlando [23] approaches is 0.002, 0.001, 0.006 and 0.006 better than ours, correspondingly. The experimental segmentation results on the STARE and DRIVE datasets confirms that the suggested method is very effective as compared to other cited frameworks. Figs 11 and 12 show visual analyses of retinal vessel extraction employing the STARE and DRIVE databases.

**Fig 11:** Visual appearance of the proposed technique utilizing STARE dataset. (a) RGB photograph (b) Manual segmentation (c) Proposed technique segmented image.

**Fig 12:** Visual appearance of the proposed technique utilizing DRIVE dataset. (a) RGB photograph (b) Manual segmentation (c) Proposed technique segmented image.

The most important aspect of suggested technique is an intelligent suppression of wrongly classified pixels clusters. Table 4 demonstrates the performance evaluation of the proposed system in case of abnormal images on the STARE database. Experimental outcomes vividly validate that for anomalous cases, the proposed system attain much better accuracy than Chaudhuri [24], Mendonça [27], Hoover [25] and Soares [15], except Lam [19] which is better than ours. Figs 13 and 14 show the visual inspection of the unhealthy fundus photographs on the STARE and DRIVE datasets, correspondingly.

**Fig 13:** Pictorial representation for unhealthy retinal image from the STARE dataset. (a) RGB image (b) Manual segmentation (c) Proposed scheme final result.

**Fig 14:** Pictorial representation for unhealthy retinal image from the DRIVE dataset. (a) RGB image (b) Manual segmentation (c) Proposed scheme final result.

**Table 4:** Proposed system segmentation results assessment with different retinal extraction approaches for abnormal retinal images.

Image Type	Method	TPR	FPR	Acc
Healty	Human observer	0.965	0.0764	0.928
	Chaudhuri [24]	0.734	0.0218	0.949
	Mendonça and Campilho [27]	0.726	0.0209	0.949
	Hoover [25]	0.677	0.0338	0.932
	Soares [15]	0.755	0.0188	0.954
	**Proposed**	**0.807**	**0.0391**	**0.964**
Anomalous	Human observer	0.825	0.0456	0.943
	Chaudhuri [24]	0.588	0.0384	0.928
	Mendonça and Campilho [27]	0.673	0.0331	0.939
	Hoover [25]	0.674	0.0528	0.921
	Soares [15]	0.687	0.0318	0.942
	Lam [19]	—	—	0.956
	Roychowdhury [21]	—	—	0.945
	**Proposed**	**0.721**	**0.0472**	**0.949**

### VLM analysis

Retinal vessel segmentation has been a hot area for research in the current decade. Although many techniques with promising results for retinal vessel segmentation have been developed but still there are some open issues particularly related to abnormal retina image and time complexity which needs to be solved in future. The future research must be accurately truthful, quicker and fully automated for retina images vessel segmentation produced by different fundus cameras. Accuracy along with sensitivity is the most significant aspect of any segmentation method and it can be enhanced by incorporating strong preprocessing and an intelligent postprocessing techniques for the rejection of incorrectly classified vessel pixels. The proposed technique has been employed on the above mentioned strategy and encouraging results have been attained. The results can be easily improved by removing exudates or pathological objects before enhancement because it is not only difficult but almost impossible to remove pathological objects after vessels enhancement stage. The effect of VLM on healthy and unhealthy retinal images are shown in Fig 15.

**Fig 15:** Proposed system results with and without using VLM on pathological (first two rows) and normal (last two rows) images from the STARE dataset. (a) Color image (b) Manual Segmented image (c) Proposed system final image without VLM (d) Segmentation results with utilizing VLM.

### Time computation

The proposed system also shows excellent performance in the case of time complexity as exposed in Table 5.

**Table 5:** Time complexity assessment of various methods with the proposed method.

Technique	Computation Time	Hardware Specifications	Software
Mendonça [27]	2.5 to 3 mins	Pentium-4, 3.2 GHz, 960 Mb RAM	MATLAB
Soares [15]	2mins (9hrs for training)	PC(2167 MHz clock), 1-GB memory	MATLAB
Lam [19]	13 mins	Duo CPU 1.83 GHz, 2.0 GB RAM	MATLAB
Staal [14]	15 mins	Pentium-III PC, CPU 1.0 GHz, 1-GB RAM	not available
**Proposed**	4.56 Sec	Core i3 CPU, 2.53 GHz, 4 GB RAM	MATLAB
Zhao [34]	22 Sec	Core i3 CPU, 3.1 GHz, 8 GB RAM	MATLAB, C

## Conclusion

The proposed technique has exhibited excellent performance as compared to other recent strategies in term of accuracy, sensitivity, specificity, FPR, TPR and AUC performance metrics. The proposed approach has performed unsupervised classification and its visual and tabulated results have evidently displayed superior performance over both supervised and unsupervised methods. Moreover, the proposed methodology has less time complexity than other existing methods. Visual results show that the proposed technique can delineate both thin and wide vessels precisely, attaining an average accuracies of 95.1%, 95.8% and 95.2% for the STARE, DRIVE and HRF datasets, respectively. Moreover, the proposed technique does not require any manual labeled information for training. That’s why it is computationally very fast and efficient also.

## Supporting information

S1 File DRIVE.zip, dataset used to test the algorithm. (ZIP)

S2 File STARE Dataset.tar, dataset used to test the algorithm. (TAR)

S3 File HRF Dataset.rar, dataset used to test the algorithm. (RAR)
